The article "Prevalence and Relevance of Multiple Renal Arteries: A Radioanatomical Perspective" was published in 2021. Journal: Cureus.

# Prevalence and Relevance of Multiple Renal Arteries: A Radioanatomical Perspective

**DOI:** 10.7759/cureus.18957

**Published:** 2021-10-21

**Authors:** Girish Pradhay, Geetha S Gopidas, Sreekumar Karumathil Pullara, Georgie Mathew, Asha J Mathew, Tintu T Sukumaran, Nanditha Pavikuttan, Rathi Sudhakaran

**Affiliations:** 1 Anatomy, Malabar Medical College Hospital and Research Centre, Calicut, IND; 2 Anatomy, All India Institute of Medical Sciences, Bibinagar, Hyderabad, IND; 3 Radiology, Amrita Institute of Medical Sciences, Amrita Vishwa Vidyapeetham, Kochi, IND; 4 Urology, Amrita Institute of Medical Sciences, Amrita Vishwa Vidyapeetham, Kochi, IND; 5 Anatomy, Amrita School of Medicine, Amrita Institute of Medical Sciences, Amrita Vishwa Vidyapeetham, Kochi, IND; 6 Anatomy, Amrita School of Medicine , Amrita institute of Medical Sciences, Amrita Vishwa Vidyapeetham, Kochi, IND; 7 Anatomy, Amrita School of Medicine , Amrita Institute of Medical sciences, Amrita Vishwa Vidyapeetham, Kochi, IND

**Keywords:** triple renal artery, double renal artery, mdct angiograms, renal artery variants, multiple renal artery

## Abstract

Background: A single renal artery supplies the kidney in 70% of the population but variation exists in the remaining 30%. Multiple renal arteries (MRA) in different permutations and combinations are one of the many forms of variants. Lack of awareness of multiplicity could have detrimental effects on the outcome of renal surgery. The present study aims at identifying the variants of renal artery based on its origin, multiplicity, and portal of entry in a cohort of people belonging to Southern India and its clinical implications thereof.

Methods: Multi-detector CT (MDCT) images of renal vasculature of 100 kidneys from 50 live kidney donors who attended the Department of Nephrology of our institution, from 2016 to 2018 were collected and studied for variations in renal arterial anatomy.

Results: Out of the 18% of kidneys observed with multiple renal arteries, 88.8% had double renal arteries (DRA) and 11.1% had triple renal arteries (TRA). Common types of the double renal arteries were - two hilar arteries (31.3%) and one hilar with one inferior polar artery (IPA, 31.3%). Triple renal arteries types - 50% with one hilar, one superior polar, and one inferior polar; 50% with two hilar and one inferior polar artery. No statistically significant association was noted between the incidence of multiple renal arteries and its laterality (p-value=0.193).

Conclusion: A thorough understanding of the renal artery variants is crucial for safe and efficacious uro-radiological interventional procedures.

## Introduction

The kidney derives its arterial supply through a single renal artery (SRA) which originates from the abdominal aorta at the level of the intervertebral disc between L1 and L2. It enters the renal hilum in relation to the renal vein anteriorly and the renal pelvis posteriorly. At or near the hilum, the renal artery divides into anterior and posterior divisions. Each division gives rise to segmental arteries within the renal sinus which supplies specific segments of renal tissue. Thus, the segmental arteries are essentially end arteries [1]. Accidental damage or ligation during surgical procedures will result in infarction of the segment supplied by it [2].

The level of origin of the renal artery may vary between T12 and L2. The atypical origin may occur from common iliac, superior mesenteric, inferior mesenteric, spermatic, ovarian, right colic, or even from the contralateral renal artery. Such arteries are referred to by different terms like, ‘aberrant’, ‘abnormal’, ‘accessory’, ‘additional’, ‘extra’, ‘supernumerary’, and ‘supplementary’. Literature consolidates these variants as ‘multiple’ to highlight the clinical significance of these vessels as separate vascular entities [3-5]. Multiple renal arteries (MRA) are present in 20-30% of individuals (two in 22%, three in 1-2%, four in 0.1%) [6]. Felix et al. in his study explained the existence of MRA embryologically [7].

Sampaio and Passos [8] classified the renal arteries based on their portal of entry into: the Hilar artery - a branch from the aorta that penetrates the kidney in the hilum; extra-hilar artery - a renal artery from the abdominal aorta which has an extra-hilar branch to the poles; superior polar artery (SPA) - a branch from the aorta that penetrates the kidney in the superior pole; inferior polar artery (IPA) - a branch from the aorta that penetrates the kidney in the inferior pole.

The nomenclature proposed by them continued to be used by subsequent researchers for classifying the renal arteries [3,9,10]. Multiplicity is very commonly noted in renal arteries than any other arteries of the same size [8,10]. With the advent of technology, CT and MRI reconstructed images of arteries, veins, and parenchyma of kidneys have added clarity in the identification of their location and structure. Insight into the existence of MRA will help prevent accidental damage per-operatively and resultant infarction of the involved segment. This has facilitated surgical planning and bettered outcomes. The present study aims to assess the incidence of anatomical variants of renal artery based on its origin, multiplicity, and portal of entry from reconstructed multi-detector CT (MDCT) images and also to find if any association exists between the type of the variant renal artery and laterality of its occurrence.

## Materials and methods

Study design and setting

A cross-sectional study was conducted for two years from 2016 to 2018. The list of 50 potential kidney donors who attended the Department of Nephrology, of our Institution, was collected for this study. The study was conducted after getting approval from the Institutional Ethical Committee (IRB- Amrita Institute of Medical Sciences, IRB-AIMS-2017-128).

Inclusion and exclusion criteria

At the donor selection stage, subjects with a previous history of renal pathology, renal transplantation, or kidney donation were excluded. The MDCT images of potential live kidney donors who had undergone a pre-operative evaluation were included in the study.

Data collection methods and tools

The MDCT images of renal vasculature of these 100 donor kidneys were accessed from the software data bank of our institution. The images were reconstructed three-dimensionally and read under the guidance of an experienced radiologist and urologist in Philips workstations.

Data analysis

The origin, multiplicity, and portal of entry of renal arteries were recorded. The variants were tabulated based on the gold standard of reference, proposed by Sampaio and Passos [8].

Sample size

Based on the study of Budhiraja et al. [9] where the percentage of MRA observed was 54.7% and with 95% confidence and 20% allowable relative error, a minimum sample size of 80 would suffice. However, the present study included 100 kidneys from 50 subjects.

Statistical analysis

The analysis was done with IBM SPSS Statistics 20.0 Windows (IBM Corp., Armonk, NY). The results are given in frequency (percentage) for categorical variables. A Chi-square test with continuity correction was applied to find the association between the types of the renal artery and the laterality. Statistically significant difference was considered if the p-value is <0.05.

## Results

In all 100 kidneys, renal arteries originated from the abdominal aorta. SRA was seen in 82 kidneys while MRA was seen in 18. Among the 18, double renal arteries (DRA) were noted in 16 (88.8%) and triple renal arteries (TRA) in 2 (11.2%). In 76 out of the 82 SRA (92.7%), the portal of entry of the renal artery was through the hilum. In three out of the 82 (3.7%), the SRA before entering the hilum gave two extrahilar branches, one to the superior pole and one to the inferior pole (Figure 1).

**Figure 1:** MDCT volume-rendered image showing SRA arising from abdominal aorta - hilar with superior pole and inferior pole extrahilar branches on both sides (anterior view) SRA: single renal artery, AA: abdominal aorta, H: hilum, CH: common hepatic artery, Sp: splenic artery, RRA: right renal artery, LRA: left renal artery, RSPEx: right superior pole extrahilar branch, LSPEx: left superior pole extrahilar branch, RIPEx: right inferior pole extrahilar branch, LIPEx: left inferior pole extrahilar branch.

In two cases (2.4%), it gave an extrahilar branch to the inferior pole whereas in one case (1.2%), it gave an extrahilar branch to the superior pole (Table 1). Among the 16 cases of DRA, five (31.3%) had an entry of both renal arteries through the hilum (Figure 2).

**Table 1:** Distribution of types of renal arteries in the present study SRA: single renal artery, MRA: multiple renal arteries, DRA: double renal arteries, TRA: triple renal arteries

Type of renal artery		Types according to the portal of entry	Total	Right kidney	Left kidney
SRA (82/100)		One hilar artery	76	40	36
		Hilar with superior pole extrahilar branch	1	1	-
		Hilar with inferior pole extrahilar branch	2	1	1
		Hilar with superior pole and inferior pole extrahilar branches	3	2	1
MRA (18/100)	DRA (16/100)	Two hilar arteries	5	2	3
		One hilar with one superior polar artery	3	1	2
		One hilar with one inferior polar artery	5	-	5
		One superior polar and one inferior polar artery	2	2	-
		Two hilar with one superior pole and one inferior pole extrahilar branches	1	1	-
TRA (2/100)		One hilar with one superior polar and one inferior polar artery	1	-	1
		Two hilar with one inferior polar artery	1	-	1

**Figure 2:** MDCT volume-rendered image showing DRA arising from abdominal aorta - hilar type on the right side (lateral view) DRA: double renal artery, AA: abdominal aorta, H: hilum, RRA1: right renal artery 1, RRA2: right renal artery 2

In five other instances (31.3%), one artery entered through the hilum, and the other entered through the inferior pole (Figure 3).

**Figure 3:** MDCT volume-rendered image showing, right side-SRA of hilar type, left side-DRA of hilar with the inferior polar type (anterior view) SRA: single renal artery, DRA: double renal artery, AA: abdominal aorta, H: hilum, RRA: right renal artery, LRA: left renal artery, LIPA: left inferior polar artery

In three cases (18.7%), one artery entered through the hilum and the other through the superior pole. In another two cases (12.5%), one renal artery entered through the superior pole and another through the inferior pole. In only one situation both the renal arteries entered through the hilum but prior to their entry, one gave an extrahilar branch to the superior pole and the other one gave an extrahilar branch to the inferior pole (Table 1).

Among the two cases of TRA, one (50%) presented with three portals of entry - first through the superior pole, second through the hilum, and third through the inferior pole. In the second case (50%), two renal arteries entered through the hilum while the third entered through the inferior pole. Table 1 classifies and summarizes the findings; 44 out of 50 right kidneys (88%) and 38 out of the 50 left kidneys (76%) presented with SRA.

Six out of 50, (12%) right-sided kidneys and 12 out of 50, (24%) left-sided kidneys presented with MRA. The association between the incidence of MRA and the side of its occurrence showed an insignificant p-value (0.193). Among the MRA, DRA was seen in six out of 50 (12%) right-sided kidneys and 10 out of 50 (20%) left-sided ones. TRA is seen only in two out of 50 (4%) left-sided kidneys. 

## Discussion

Normally, a single renal artery originating from the abdominal aorta divides at the hilum to give anterior and posterior divisions which enter the kidney. But it is not very uncommon to see one or more extra or accessory arteries entering the renal tissue to supply it. An extensive study on the types of accessory renal arteries, their positions, method of entry, and the branching pattern was done by Sykes [9]. Studies have shown that these extra arteries entering the kidney through the hilum or the poles are end arteries supplying a particular renal segment. As there is no collateral circulation between the segments, damage of such arteries may lead to ischaemia and necrosis of that particular segment supplied by them [11]. So they cannot be considered as ‘extra’ or ‘accessory’. They are indeed essential arteries that are equivalent to segmental branches of SRA. According to Sampaio and Passos, they should be grouped as MRA. Sampaio and Passos analysed the renal vasculature of 266 kidneys by dissection and reported a single hilar artery in 53.3%; one hilar artery with one superior polar extra-hilar branch in 14.3%; double hilar artery in 7.9%; one hilar with one SPA in 6.8%; one hilar with one inferior polar artery in 5.3%; two hilar with one superior pole extra-hilar branch in 3.4%; triple hilar artery in 1.9% and other variation in 8.5% [8].

The embryological basis of the existence of MRA was proposed by Felix et al. in 1912. According to him, in an 18 mm fetus, mesonephros, metanephros, suprarenal glands, and gonads receive blood supply from nine pairs of lateral mesonephric arteries which are arising from the dorsal aorta. He categorized these arteries into three: cranial (first and second), middle (third to fifth), and caudal (sixth to ninth). A single pair from the middle group develops into the renal artery normally. Any other artery persisting from these groups will exist as the variant MRA [7].

In the present study, out of the 18 cases of MRA, 12 belonged to the left side. A higher prevalence of MRA on left was reported by several authors [2,12-14]. Budhiraja et al. observed a high incidence of MRA (54.7%), more on the right side [9]. The literature says about 30% of normal subjects may have MRA while the incidence may range from 11% to 61% [15]. Literature states that the occurrence of MRA may vary with ethnicity [8,12,15-18].

Bordei et al. noted that additional renal arteries entered through the hilum of the kidney in 61.11% of cases, through the superior pole in 9.26%, and through the inferior pole in 29.63% [12]. We observed a low range of variability as compared to the data furnished by Budhiraja et al. in the population of Central India [9] (Table 2).

**Table 2:** Comparison of incidence of multiple renal arteries in different population groups DHA: double hilar artery, THA: triple hilar artery, SPA: superior polar artery, IPA: inferior polar artery

Authors	Year	Population	DHA	THA	SPA	IPA
Sampaio and Passos [8]	1992	Caucasians	7.90%	1.90%	6.80%	5.30%
Ciçekcibaşi et al. [19]	2005	Turkish	11.10%	-	3.30%	10.50%
Weld et al. [20]	2005	American	12.30%	-	9.60%	15.10%
Talovic et al. [21]	2007	Bosnian	9%	1%	2%	10%
Guan et al. [22]	2011	Brazilian	45.50%	18.80%	9.40%	3.20%
Budhiraja et al. [9]	2012	Indian	22.60%	11.80%	13.10%	7.10%
Present study		Indian	7%	-	6%	9%

The incidence of MRA may vary in the same geographical region itself depending on the differences in environmental factors that influence the organogenesis period [12].

In the present study, we observed branches of renal arteries penetrating extrahilar renal tissue and compared its percentage distribution with the previous study. The extrahilar portal of entry is more frequent on the right side which is comparable to the data given by Budhiraja et al. [9] and Talovic et al. [21] (Table 3).

**Table 3:** Percentage distribution of extrahilar branch of renal artery for the right and the left kidney in different population groups

Authors	Year	Extrahilar superior polar		Extrahilar inferior polar	
		Right kidney	Left kidney	Right kidney	Left kidney
Talovic et al. [21]	2007	10%	2%	2%	0
Palmieri et al. [22]	2011	28.60%	11.60%	0	1.40%
Budhiraja et al. [9]	2012	21.40%	19%	11.90%	2.40%
Present study		8%	2%	8%	4%

Guan et al. [22] and Bordei et al. [12] reported that the accessory inferior polar arteries are the most common type of MRA. Inferior polar artery (IPA) has greater clinical relevance than SPA as the upper part of the ureter is supplied by a branch of IPA if it exists. Damage to this vessel will result in ureteric necrosis leading to paralysis or urinary leak [10]. It could constrict the ureter at the ureteropelvic junction as it traverses anterior or posterior to it, leading to hydronephrosis [23]. Extrahilar superior and inferior polar arteries may get injured during mobilization and other surgical procedures on the renal poles [8].

Unusual origins of variants were observed from several arteries such as - external iliac, median sacral, splenic, lumbar, superior suprarenal, inferior phrenic, thoracic aorta, etc. [24]. But in the present study, we noted the origin of renal arteries to be only from the abdominal aorta.

Kidneys with SRA are preferred for renal transplantation but it is technically acceptable to transplant a kidney with MRA [25].To be kept in mind is that transplant that involves MRA can have increased morbidity due to the risk of complications like haemorrhage, infarction, arterial thrombosis, longer operating time, stenosis at suture lines, and graft failure [26].

Assessment of arterial anatomy of the kidney is mandatory for preoperative evaluation in renal transplantation, implantation of renal arterial stents in reno-vascular hypertension, vascular reconstruction, etc. [27]. This study is an attempt to enrich the compendium of knowledge and thereby ultimately improve awareness regarding the multiplicity of renal arteries. This will go a long way in reducing the risk of surgical failure and postoperative complications.

## Conclusions

The origin and number of multiple renal arteries are complex occurrences. These arteries can be considered embryologically relevant, attributable to a failure to degenerate during the ascent of the metanephros in search of a higher pressure head. The frequency can be as high as 30% of the population. The present study observed different types of anatomical variations of renal arteries. The presence of multiple renal arteries is the most important among them. A thorough awareness of the possibilities of distribution of MRA will help the surgeon to perform the surgeries on kidney and renal transplantation more effectively.
